# Emergence of Asian endemic begomoviruses as a pandemic threat

**DOI:** 10.3389/fpls.2022.970941

**Published:** 2022-09-28

**Authors:** Muhammad Amir Qureshi, Aamir Lal, Muhammad Shah Nawaz-ul-Rehman, Thuy Thi Bich Vo, Gusti Ngurah Prabu Wira Sanjaya, Phuong Thi Ho, Bupi Nattanong, Eui-Joon Kil, Shah Mohammad Hemayet Jahan, Kyeong-Yeoll Lee, Chi-Wei Tsai, Hang Thi Dao, Trinh Xuan Hoat, Tin-Tin Aye, Nang Kyu Win, Jangha Lee, Sang-Mok Kim, Sukchan Lee

**Affiliations:** ^1^Department of Integrative Biotechnology, Sungkyunkwan University, Suwon, South Korea; ^2^Centre of Agricultural Biochemistry and Biotechnology, University of Agriculture, Faisalabad, Pakistan; ^3^Department of Plant Medicals, Andong National University, Andong, South Korea; ^4^Department of Entomology, Patuakhali Science and Technology University, Dhaka, Bangladesh; ^5^Division of Applied Biosciences, College of Agriculture and Life Sciences, Kyungpook National University, Daegu, South Korea; ^6^Department of Entomology, National Taiwan University, Taipei, Taiwan; ^7^Plant Protection Research Institute, Hanoi, Vietnam; ^8^Department of Entomology, Yezin Agricultural University, Yezin, Myanmar; ^9^Department of Plant Pathology, Yezin Agricultural University, Yezin, Myanmar; ^10^Crop Breeding Research Center, NongWoo Bio, Yeoju, South Korea; ^11^Plant Quarantine Technology Center, Animal and Plant Quarantine Agency, Gimcheon, South Korea

**Keywords:** Asia, geminiviruses, begomoviruses, geographical distribution, Tomato leaf curl New Delhi virus, Papaya leaf curl virus, Tomato yellow leaf curl virus

## Abstract

Plant viruses are responsible for the most devastating and commercially significant plant diseases, especially in tropical and subtropical regions. The genus *begomovirus* is the largest one in the family *Geminiviridae,* with a single-stranded DNA genome, either monopartite or bipartite. Begomoviruses are transmitted by insect vectors, such as *Bemisia tabaci*. Begomoviruses are the major causative agents of diseases in agriculture globally. Because of their diversity and mode of evolution, they are thought to be geographic specific. The emerging begomoviruses are of serious concern due to their increasing host range and geographical expansion. Several begomoviruses of Asiatic origin have been reported in Europe, causing massive economic losses; insect-borne transmission of viruses is a critical factor in virus outbreaks in new geographical regions. This review highlights crucial information regarding Asia’s four emerging and highly destructive begomoviruses. We also provided information regarding several less common but still potentially important pathogens of different crops. This information will aid possible direction of future studies in adopting preventive measures to combat these emerging viruses.

## Introduction

Geminiviruses are the most destructive group of viruses infecting agricultural crops in the tropical and subtropical regions of the world (Laufs et al., 1995; Mansoor et al., 2003; Marwal et al., 2012; Inoue-Nagata et al., 2016). They are also among the largest group of viruses transmitted by whiteflies (*Bemisia tabaci*; Bedford et al., 1994; Inoue-Nagata et al., 2016). The members of family *Geminiviridae* have circular single-stranded DNA (ssDNA) genome encapsulated in a twinned icosahedral coat protein.

In the nineteenth century, symptoms of geminivirus infection were first observed in plants in the tropical and subtropical regions (Moffat, 1999; Inoue-Nagata et al., 2016; Orfanidou et al., 2019). They seriously threatened crop production and agricultural fields (Moffat, 1999). However, in this century, multiple newly emerging geminiviruses have destroyed crops, such as legumes, cotton, and tomatoes (Cohen and Antignus, 1994; Varma and Malathi, 2003). For example, in Africa, the geminiviruses on cassava plants caused an economic loss of approximately US$ 1,300–2,300 million (Hillocks et al., 2002), and in the United States, the tomato yellow leaf curl disease (TYLCD) resulted in an average loss of US$ 140 million every year (Morales and Anderson, 2001).

### Geminivirus strains and species

The International Committee on Taxonomy of Viruses group working on the family *Geminiviridae* proposed a new standard for species identification (Francki et al., 2012). Based on this classification, more than 500 geminiviruses have been distinguished and characterized into 14 distinct genera (Chiumenti et al., 2021; Lal et al., 2021). The order of various genera depends on the genome, host range, and viral vectors (Fauquet et al., 2003; Varsani et al., 2014). Currently recognized genera of *Geminiviridae*, their properties, and type members are described in Table 1. Figure 1 depicts the species distribution in each genus.

**Table 1:** Currently recognized genera of the *Geminiviridae*, their properties, and type members by ICTV.

Genus	Insect vector	Genome	Host	Member species	References
*Begomovirus*	*B. tabaci*	Monopartite /Bipartite	Monocots/Dicots	*Bean golden mosaic virus*	Brown et al., 2015
*Eragrovirus*	Unknown	Monopartite	Monocots	*Eragrostis curvula streak virus*	Varsani et al., 2014
*Becurtovirus*	*Circulifer haematoceps*	Monopartite	Dicots	*Beat curly top Iran virus*	Claverie et al., 2018
*Mastrevirus*	*Cicadulina mbila*	Monopartite	Monocots	*Maize streak virus*	Muhire et al., 2013
*Topocovirus*	*Micrutalis malleifera*	Monopartite	Dicots	*Tomato pseudo-curly top virus*	Briddon et al., 1996
*Grablovirus*	*Spissistilus festinus*	Monopartite	Eudicots	*Grapevine red blotch virus*	Krenz et al., 2012
*Capulavirus*	*Aphis craccivora*	Monopartite	Dicots	*Euphorbia caputmedusae latent virus*	Bernardo et al., 2013
*Turncurtovirus*	*Cicadellidae*	Monopartite	Dicots	*Turnip curly top virus*	Varsani et al., 2014
*Curtovirus*	*Circulifer tenellus*	Monopartite	Dicots	*Beet curly top virus*	Stanley et al., 1986
*Citlodavirus*	*Aphis gossypii*	Monopartite	Dicots	*Citrus chlorotic dwarf associated virus*	Loconsole et al., 2012
*Maldovirus*	unknown	Monopartite	Both	*Apple Geminivirus 1*	Liang et al., 2015
*Mulcrilevirus*	*Tautoneura mor*	Monopartite	Monocots	*Mulberry crinkle leaf virus*	Lu et al., 2015
*Opunvirus*	*Cochineal insects*	Monopartite	Dicots	*Opuntia virus 1*	Fontenele et al., 2020
*Topilevirus*	*Micrutalis malleifera*	Monopartite	Dicots	*Tomato apical leaf curl virus*	Vaghi Medina et al., 2018

**Figure 1:** Species distribution of geminivirus. Number of species in each genus. It can be clearly seen that the genus *Begomovirus* has the highest number of species among the family *Geminiviridae.*

### General characteristics of begomoviruses

The largest and most important genus of *Geminiviridae* is *Begomovirus*, transmitted by the whitefly (*B. tabaci*): (Khan et al., 2012; Yaqoob et al., 2020; Vivek et al., 2021). It is proposed that single stranded DNA viruses developed from prokaryotic episomal DNA and recombine with the target plant’s genome to acquire new characteristics (Rojas et al., 2005). The size of the begomovirus genome is between 2,600 and 2,800 nucleotides (Ho et al., 2014). They replicate by rolling circle amplification (RCA) using a double-stranded DNA (dsDNA) intermediate (Yadava et al., 2010). Begomoviruses are classified into four categories based on their genomic structure and evolutionary relationships: New World (NW), Old World (OW), Sweepoviruses, and Legumoviruses (Fiallo-Olivé et al., 2021). In OW and NW, pepper, tomato, and cucurbit plants are common hosts for begomoviruses (Seal et al., 2006). Most NW begomoviruses have a bipartite genome made up of DNA-A and DNA-B components. DNA-A found both in monopartite and bipartite begomoviruses, they are similar from genomic structure and arrangement point of view and have similar proteins encoding genes like C1/AC1, C2/AC2, C3/AC3, C4/AC4, C5/AC5 and V1/AV1 (Gutierrez, 1999; Harrison and Robinson, 1999; Zhao et al., 2022). They also have V2 protein which is absent in OW bipartite begomoviruses. But NW bipartite has AV2 genes analogue to this V2 gene of monopartite (Sudarshana et al., 1998; Rojas et al., 2005). V3 protein is also present, essential for complete viral infection and works as an RNA silencing suppressor (Gong et al., 2021). DNA-B is found in bipartite genome. It interprets two proteins for cell-to-cell movement (Briddon et al., 2010). Two proteins are BV1 and BC1. It also has Intergenic region (IR). IR has a region named as conserved region in which about 200 nucleotides are there which carry almost sequence similarity of more than 85%. This has nonanucleotide sequence which is found in all geminiviruses, and it is their speciality (Roshan et al., 2017). Begomoviruses in the OW can be both monopartite or bipartite and are associated with betasatellites, alphasatellites and deltasatellites (Fiallo-Olivé et al., 2021). Alphasatellites, which are mostly found in monopartite OW begomoviruses, have a genome that encodes a replication-associated protein that is required for replication. Betasatellites, which are found in association with many monopartite OW begomoviruses, are required for the onset of common disease symptoms (Zhou, 2013; Gnanasekaran et al., 2019). The betasatellite genome encoded C1 protein plays vital functions in symptom induction and the inhibition of transcriptional and post-transcriptional gene silencing (Li et al., 2018). Deltasatellites, unlike betasatellites and alphasatellites, do not encode any gene. All deltasatellites share several genomic features, including a stem-loop containing the conserved begomovirus nonanucleotide TAATATTAC, a putative secondary stem-loop structure located near begomovirus iteron-like sequences, a short region with the sequence identity of the betasatellite conserved region, and an A-rich region (Fiallo-Olivé et al., 2012). NW bipartite begomoviruses have also potential to interact with betasatellite. Cotton leaf curl Multan betasatellite (CLCuMuB) associated with a serious disease of cotton is capable to interact with NW begomovirus. NW Cabbage leaf curl virus of interact with CLCuMuB to enhanced symptoms development in *Nicotiana Benthamiana* (Nawaz-ul-Rehman and Fauquet, 2009). Figure 2 depicts the genomic structure of the begomovirus.

**Figure 2:** Begomovirus genome: **(A)** DNA-A segment of begomovirus. **(B)** DNA-B segment found in bipartite begomovirus along with DNA-A. **(C)** Alphasatellite, **(D)** betasatellite and **(E)** deltasatellite associated with monopartite begomoviruses.

### Host range and symptoms

Begomovirus infects a wide range of dicot and monocot plants and causes severe loss, exhibiting symptoms such as stunting, deformed growth, and decreased seed production in infected plants (Dasgupta et al., 2003); leaf crumpling, curling, distortion, golden-light green-yellow mosaic/mottle, interveinal yellowing, yellow spots, vein swelling, purpling, and yellowing in dicotyledonous plants (Rishi, 2009). Table 2 describes the host range and symptoms of some important begomoviruses.

**Table 2:** Host range and symptoms of certain destructive begomoviruses in the world.

Name	Host range	Symptoms	References
*Cotton leaf curl Multan Virus*	*Gossypium hirsutum*, Hibiscus *rosa-sinensis, H. esculentus*, *Malvaviscus arboreus*, *Gossypium hirsutum*, and H*. cannabinus*	Downward and upward curling of leaves, vein thickening, and yellowing	Rahman et al., 2017
*Papaya leaf curl China virus*	*Nicotiana tabacum, Carica papaya, Solanum lycopersicum, Corchoropsis timentosa, Sigesbeckia orientalis, A. conyzoides, Acalypha australis*	Severe curling, crinkling, and rolling of leaves	Zhang et at., 2010
*Sweet potato leaf curl virus*	*Ipomoea batatas* (L.), *Ipomoea setosa, Ipomoea wrightii*	Chlorosis, yellowing, curling, and stunting	Paprotka et al., 2010
*Tomato yellow leaf curl virus*	*Solanum lycopersicum, Vigna unguiculata, Phaseolus vulgaris, Solanum melongena*	Leaf chlorosis, curled-up margins, and stunted growth	Khan et al., 2013
*Euphorbia leaf curl virus*	*Euphorbia pulcherrima, Carica papaya, Nicotiana sp., Solanum lycopersicum, Petunia hybrid, Datura stramonium*	Yellow, curling of leaves, and vein thickening	Tsai and Huang, 2017
*Mungbean yellow mosaic virus*	*Glycine max, Phaseolus vulgaris, Vigna mungo, Glycine max, Cajanus cajan*	Mosaic and slightly stunting symptoms	Mishra et al., 2020
*Tobacco leaf curl Geminivirus*	*Nicotiana tabacum, Solanum lycopersicum, Spinacia oleracea, Lonicera japonica, Capsicum annuum*	Vein yellowing, enations, and leaf curling	Jing et al., 2016
*Tomato leaf curl Joydebpur Virus*	*Solanum lycopersicum, Capsicum frutescens, Phaseolus vulgaris, Solanum nigrum, Amaranthus viridis, Hibiscus*	Yellowing, shrinking of leaves, severe leaf curling, and extra dwarfing	Hamim et al., 2020
*Ageratum yellow vein virus*	*Ageratum conyzoides, Petunia x hybrida, Sauropus androgynus*	Leaf curling, yellowing, vein thickening, puckering, small leaves, and stunting	Kesumawati et al., 2020
*Tomato leaf curl New Delhi virus*	*Solanum lycopersicum, Solanum melongena, Cucumis melo, Cucumis sativus, Cucurbita pepo Capsicum, Solanum tuberosum, Cucurbita*	Leaf curling and yellow mosaic	Hamim et al., 2020

### Geminiviruses are unequally distributed across the continents

The Geminiviruses are present on all the continents except Antarctica. Maximum diversity of geminiviruses exists in Southeast Aisa. In contrast to several tropical and subtropical regions, the genetic variability of *Geminiviridae* in Europe is low (Bendahmane et al., 1995; Lindsten and Lindsten, 1999). Wheat dwarf virus, a solitary *Mastrevirus* localized to northern and central Europe, causes scattered yield loss in wheat (Bendahmane et al., 1995; Lindsten and Lindsten, 1999). All other geminiviruses found in Europe belong to the genus *Begomovirus* and are distinguished based on their genetic characteristics and region of origin (Briddon, 2002). Table 3 lists some crucial begomoviruses on the European and Mediterranean Plant Protection Organization (EPPO) alert list. Tomato yellow leaf curl virus (TYLCV) and Tomato leaf curl New Delhi virus (ToLCNDV) are prominent begomoviruses in Europe, which were previously limited to Mediterranean and Indian subcontinent respectively.

**Table 3:** EPPO alert list of important begomoviruses from 2000 to 2021.

Viruses	Hosts (First identified)	Hosts (All reported)	2000–2021
*Tomato yellow mosaic begomovirus*	*Solanum tuberosum*	*Solanum lycopersicum, Solanum pimpinellifolium*	2000
*Abutilon mosaic virus*	*Gossypium hirsutum*	*Abutilon hybrids, Malvaceae*	2000
*Chino del tomato virus*	*Solanum lycopersicum*	*Capsicum annuum*	2001
*Pepper huasteco yellow vein virus*	*Capsicum annuum*	*Cucumis sativus, Solanum lycopersicum*	2001
*Pepper mild tigre virus*	*Capsicum annuum*	*Solanum lycopersicum*	2001
*Pepper golden mosaic virus*	*Solanum lycopersicum*	*Capsicum annuum, Capsicum frutescens, Nicotiana tabacum*	2001
*Tomato yellow vein streak virus*	*Solanum lycopersicum*	*Solanum tuberosum*	2001
*Potato yellow mosaic virus*	*Solanum tuberosum*	*Lycopersicon esculentum*	2003
*Bean golden mosaic virus*	*Phaseolus vulgaris*	*Calopogonium, Fabaceae, Phaseolus lunatus*	2004
*Tomato yellow leaf curl virus*	*Solanum lycopersicum*	*Phaseolus vulgaris*	2008–2016
*Tomato leaf curl New Delhi virus*	*Zucchini squash, cucurbit crops*	*Cucurbitaceae and Solanaceae*	2015
*Watermelon chlorotic stunt virus*	*Cucurbita moschata*	*Solanum lycopersicum, Cucumis melo, Citrullus lanatus*	2007
*Tomato dwarf leaf curl virus*	*Solanum lycopersicum*	*Capsicum annuum*	2001

### Tomato yellow leaf curl virus

*Solanum lycopersicum* (Tomato) is the host of a large number of viruses. These viruses cause significant losses in fruit production and quality (Hanssen et al., 2010). TYLCV is one of the important begomoviruses and it currently ranks third on the list of crucial plant viruses worldwide (Scholthof et al., 2011; Rybicki, 2015). The first case of TYLCD was reported in the late 1930s in Jordan Valley, Israel, and TYLCV was officially declared the virus of this disease after the 1960s (Mabvakure et al., 2016). After that, TYLCV expanded uncontrolled across the Mediterranean basin and most tropical and subtropical areas of the globe, and it is now recognized as one of the world’s most damaging virus for tomato (Lefeuvre et al., 2010). The disease continues to spread to new areas, with significant outbreaks in Trinidad and Tobago (Chinnaraja et al., 2016) and Costa Rica (Barboza et al., 2014).

TYLCV and 12 TYLCV-like viruses are members of a virus complex that causes TYLCD https://talk.ictvonline.org/taxonomy/. The significant symptoms of TYLCD in tomatoes are leaf discoloring, curling, and plant stunting. Furthermore, during extreme infection, flowers, and fruit were abscised, followed by a full reduction in plant growth. (Yan et al., 2021).

Although TYLCD spread worldwide, however, just two strains namely Mild (TYLCV-Mild) and Israel (TYLCV-IL) are truly international TYLCD-causing entities (Navas-Castillo et al., 2011). Numerous begomoviruses associated with TYLCD were found only in specific geographic areas, such as Tomato yellow leaf curl Sardinia virus and Tomato yellow leaf curl China virus, which was observed only in the Mediterranean and China (Navas-Castillo et al., 2011; Pan et al., 2012). The trading of plant materials is a significant contributor to the global spread of TYLCD (Seal et al., 2006). This global distribution is also associated with the worldwide increase in the population of insect vectors and the rapid evolution of virus variants (Mabvakure et al., 2016).

TYLCV is potentially distinctive among begomoviruses in that it can replicate within *B. tabaci* (Czosnek et al., 2017; He et al., 2020) and seeds (Kil et al., 2016; Pérez-Padilla et al., 2020) Such feature may have contributed significantly to its global distribution and is spreading to new areas in the Indian and Pacific regions, including New Caledonia, Australia, and Mauritius. A study was conducted in which they performed a temporal-scaled, phylogeographic analysis of all publicly released TYLCV complete genome sequences and 70 new genomic sequences from Australia, Iran, and Mauritius. This indicated that epidemics in Australia and China were probably the product of multiple individual viral introductions from the East Asian region surrounding Japan and Korea. The New Caledonian epidemic was due to a variant from the Western Mediterranean region, and the Mauritian outbreak by a variant from the adjacent Island of Réunion. This study also revealed that the movement of TYLCV to East Asia has stopped temporarily, while that to America and Australia continues (Mabvakure et al., 2016). The TYLCV spread in new countries after 2010 can be seen in Figure 3.

**Figure 3:** Expansion of TYLCV on the world map. Possible infected countries are highlighted in two different ways. Green dots indicate the infected countries till 2010, while red triangles indicate the expansion of this virus into new countries.

### Tomato leaf curl New Delhi virus

One of the most noticeable disease on tomatoes and other vegetables in Asia and now in Europe is the ToLCNDV (Briddon, 2002; Hussain et al., 2004). Unlike TYLCV, which is monopartite in nature, the ToLCNDV is a bipartite begomovirus that causes damage to cultivated plant species of the *Solanaceae* family, including tomato, *Solanum tuberosum* (potato), *Capsicum frutescens* (chili), *Piper nigrum* (pepper), and *Solanum melongena* (eggplant). In its early days, its outbreak was restricted to Asian countries (Moriones et al., 2017). Recently, ToLCNDV has increased its host plant range, including *Euphorbiaceae*, *Cucurbitaceae*, *Fabaceae*, and *Malvaceae* (Moriones et al., 2017).

ToLCNDV was first reported in the western Mediterranean region in 2012, infecting *Cucurbita pepo L* (zucchini squash), *Cucumis melo L* (melon), and *Cucumis sativus L* (cucumber) crops in Southern Spain (Juárez et al., 2014; San Ambrosio and Fernández, 2015). Recent ToLCNDV epidemics in the Mediterranean basin have been associated with the emergence of a new strain, ToLCNDV-ES, which primarily attacks cucurbits, such as cucumber, zucchini, and melon. The molecular characterization of this virus revealed that it had 98% similarity to partial Coat protein gene sequences from isolates of ToLCNDV, which infects cucumber plants in India (Desbiez et al., 2020). The emergence of ToLCNDV in the Mediterranean Basin poses a new threat to commercially vital cucurbit crops and tomato production, as Spain is a significant producer of cucurbits worldwide and Europe’s first exporting country (Juárez et al., 2014; Ruiz et al., 2017).

ToLCNDV was then found to infect zucchini crops in Greece in 2018 (Orfanidou et al., 2019), adding to its geographical diversity. Later, ToLCNDV expanded to Tunisia, Italy, Morocco, and Greece (Panno et al., 2016; EFSA Panel on Plant Health et al., 2020). Furthermore, ToLCNDV has recently been identified in cucurbit plants in Portugal and Estonia and in members of the *Solanaceae* family in Italy, indicating that it is rapidly spreading throughout Europe (Parrella et al., 2018, 2020). The expansion of ToLCNDV can be seen in the world map in Figure 4.

**Figure 4:** The emergence of ToLCNDV in Europe and Africa. Green dots indicate that infection was dominant in Southeast Asia until 2010. Blue triangles indicate the invasion of ToLCNDV in Europe and North Africa after 2010.

### Cotton leaf curl disease (CLCuD) in the Indian sub-continent is a major limiting factor on cotton crop

Begomoviruses pose a serious threat to all major crops in Asia, e.g., CLCuD has been observed to be caused by various begomoviruses, i.e., Cotton leaf curl Multan virus (CLCuMuV), Cotton leaf curl Kokhran virus (CLCuKoV), Cotton leaf curl Gezira virus (CLCuGV), Cotton leaf curl Burewala virus etc. (Briddon and Markham, 2000; Farooq et al., 2011). These cotton-infecting viruses may work in association with betasatellites to cause infection, i.e., CLCuMuB in Asia and cotton leaf curl Gezira betasatellite (CLCuGB) in Africa (Tahir et al., 2011).

Asia and the Mediterranean regions suffer from leaf curling disease due to the begomoviruses and satellite DNA that make up a complex system (Nawaz-ul-Rehman and Fauquet, 2009). However, they are not the same globally. Therefore, infection experiments were conducted on different groups of monopartite and satellite particles. The combinations were as follows: CLCuKoV, CLCuMuV, *okra yellow crinkle virus*, and *ageratum leaf curl Cameroon alphasatellite*. This study provides evidence for the interaction of begomoviruses with unrelated DNA satellites, which evolved new complexes of these begomoviruses in Asia. This may occur across continents, leading to the development of novel viruses (Sattar et al., 2019).

### Cassava mosaic disease can cause famine in Africa

Cassava mosaic disease (CMD)-related viruses are another example of essential begomoviruses in Africa, Sri Lanka and India. Currently, the *Manihot esculenta* (cassava) crop is highly influenced by CMD due to the activity of at least nine bipartite local African begomoviruses, called cassava mosaic geminiviruses (CMGs; De Bruyn et al., 2016). This high level of diversification indicated several local virus introduction events in this crop. Madagascar, a restricted geographical area, can serve as an example of various introduction events and interactions of this group of CMGs (De Bruyn et al., 2016). Since the late 1980s, CMGs have accelerated the spread of CMD outbreaks, damaging cassava crops in almost 12 African countries and the southwest Indian Ocean islands (Legg et al., 2011).

African cassava mosaic virus (ACMV) is the most common cassava mosaic begomovirus in Nigeria. Which spread by contaminated stem cuttings and whitefly vectors (Eni et al., 2021). Although CMD has been prevalent in Africa since the nineteenth century, it was not known in Southeast Asia until May 2015, when the first CMD epidemic was discovered in Cambodia (Wang et al., 2016). The viral species causing CMD in Southeast Asia is Sri Lankan cassava mosaic virus (SLCMV), a bipartite begomovirus that is common in Cambodia, Vietnam, Thailand, and south China (Siriwan et al., 2020).

### A global movement of begomoviruses that pose a serious threat

Emerging begomoviruses pose a serious threat to agricultural production worldwide. These viruses can be new (i.e., previously unknown) or already known; however, they share the common characteristic of occupying and spreading within new niches (Elena et al., 2014; Ertunc, 2020). The factors driving the emergence of plant viruses include genetic variability and the global movement of plant materials, i.e., nursery plantations (Rojas and Gilbertson, 2008; Elena et al., 2014). By applying modern science, improved cultivated crop varieties (“cultivars”) can significantly enhance crop yields and improve agricultural productivity. Improved cultivars can lead to greater production combined with other modern inputs and good crop management practices. This has increased the demand for improved seeds worldwide (Baker and Smith, 1966; Johansen et al., 1994; Evenson and Gollin, 2003). Therefore, the study of seed transmission of begomoviruses is crucial to limit the spread of viruses.

Several studies on the localization and movement of begomoviruses in host plant system have concluded that the virus is limited to cambium and phloem parenchyma cells of plants. Sometimes, they exit the phloem and enter the mesophyll parenchymatous tissue (Rojas et al., 2005; Rojas and Gilbertson, 2008). One advantage of horizontal virus transmission is the limited transmission of viruses among nearby plants. Compared with horizontal transmission, viruses transmitted by infected seeds can play a crucial role in viral stability from parents to offspring and between seasons (Simmons et al., 2011).

It is crucial to identify viral transmission methods, as it helps to understand the epidemiology and outbreak of viruses (Kim et al., 2015). The transmission of begomoviruses by infected seeds has been limited for many years, and viruses can only be transmitted through insects, sap, and inoculation mechanisms (Stanley et al., 2001). However, multiple begomoviruses, such as Mung bean yellow mosaic virus, TYLCV, ToLCNDV (Sangeetha et al., 2018; Kil et al., 2020), and Dolichos yellow mosaic virus, are seed-transmissible viruses (Kil et al., 2016). It was recently discovered that TYLCV could be transmitted through infected tomato seeds (Kil et al., 2016; Pérez-Padilla et al., 2020).

Transovarial transmission of viruses from vector parents to offspring is important for their epidemiology. The majority of begomoviruses are limited to transmit only by insect vector but TYLCV have been found to show transovarial transmission. It was observed that TYLCV access into the reproductive organ of its vector was mostly determined by the developmental stage of the whitefly ovary, and that TYLCV transmission to offspring increased with whitefly adult age. The precise interaction between viral coat protein with whitefly vitellogenin was required for virus entry into the whitefly ovary (Wei et al., 2017).

### Role of insect vectors

The global increase in the population of insect vectors and the rapid evolution of virus variants are also associated with the worldwide distribution of begomoviruses (Mabvakure et al., 2016). The role of insect vectors, which is the key factor in the spread of begomoviruses, also contributes to their evolution (Seal et al., 2006; Materatski et al., 2021). The adaptive response of co-evolution among viruses and insects is supported by the continual and circulative dispersal of the virus in the insect vector and the direct connection between begomoviruses and insects (Nawaz-ul-Rehman and Fauquet, 2009; Gupta et al., 2021).

*Bemisia tabaci,* is the key player in the global spread of begomoviruses. Its increased adaptability resulted in the introduction of many begomoviruses in previously unreported areas (Islam and Wu, 2017). Squash leaf curl virus, for example, was discovered in Israel in 2002 and rapidly spread to the Middle East. Some other latest examples of the global distribution of begomoviruses, which followed the invasion path of *B. tabaci,* include ToLCNDV from India to southern Spain (Hagen et al., 2008) and cucurbit leaf curl virus from the southwestern United States to Florida (Juárez et al., 2014).

### The connection between virus complexes and betasatellites

Another aspect involved in begomovirus outbreaks is the connection of complex viruses with betasatellites. In TYLCD, the first betasatellite, i.e., CLCuGB associated with either TYLCV-IL or TYLCV-Mild in tomato plants was reported in very recent times in Israel (Gelbart et al., 2020), as the Mediterranean basin and the Middle East are suggested to be hubs of both TYLCV complex root and diversification. This is a major issue for farmers globally, particularly native to the Mediterranean area. Currently, 61 betasatellite species have been reported. More than 90% of betasatellite species are found in China and the Indian subcontinent. The coordinated efforts to prevent the further spread of betasatellites into the complex’s genetic pool can restrict the emergence of begomovirus–betasatellite disease complexes.

### Recent introduction of *Cotton leaf curl Gezira virus* to the United States

Two complexes of CLCuD have been identified in the OW: the African and Asian complexes. Although CLCuD was originally identified in Africa in 1912 (Farquharson, 1912), the causal agent was not discovered until much later (Sattar et al., 2013). Only CLCuGV has been found in African cotton; however, few cotton samples have been examined, and the exact diversity of begomoviruses may be considerably greater than we currently recognize (Idris and Brown, 2002). CLCuGV is a geographically widespread virus from central Africa to Jordan that infects various plant species, including cotton, Abelmoschus esculenta (okra), Alcea (hollyhock), and Salix alba (white willow; Idris and Brown, 2002; Tahir et al., 2011).

CLCuGV-satellite complex members have lately been found in the African Sahel, Arabian Peninsula and the Middle East, Pakistan, and recently in okra in southern Texas, USA (Tiendrébéogo et al., 2010; Tahir et al., 2011; Idris et al., 2014; Villegas et al., 2019). The origin of this OW CLCuGV-satellite complex in NW okra plants is unknown; however, it was possibly introduced by diseased plant materials or virulent whiteflies brought into Southern Texas, which is known for its extensive cotton and vegetable production. The spread of this disease poses a significant threat because cotton and vegetable cultivars grown in the US have no resistance to CLCuGV (Villegas et al., 2019).

Research has shown that exotic begomoviruses can disrupt the local disease patterns of known begomoviruses. For example, the TYLCV has expanded from Asia to become the globally tomato-infecting begomovirus, including the Dominican Republic, Spain, Sicily, Italy, and Indian Ocean islands (Davino et al., 2006; Delatte et al., 2007). ToLCNDV was initially identified in North India in 1995 (Srivastava et al., 1995) and has since been reported throughout the region (Sohrab et al., 2003; Raj et al., 2005; Khan et al., 2006; Labarrere et al., 2011). Subsequently, the virus was reported in other neighboring countries, such as Pakistan (Hussain et al., 2004, 2005; Haider et al., 2006), Bangladesh (Maruthi et al., 2005), Thailand (Ito et al., 2008), Indonesia (Mizutani et al., 2011), and Spain (Juárez et al., 2014; Desbiez et al., 2020). Therefore, it is very important to study the geographical distribution of begomoviruses.

### Geographical distribution of some important begomoviruses

The growing phenomenon of begomoviruses and the attack of native viruses on crops, such as tomato, cotton, or cassava, indicates that existing outbreaks are the outcome of current begomoviruses colliding with recently launched hosts or vectors instead of dynamic changes in geminiviruses (Seal et al., 2006; Nawaz-ul-Rehman and Fauquet, 2009). Begomoviruses exploit the same whitefly vector, are extremely recombinogenic, and are widespread in tropical and subtropical areas, posing a severe threat to global food security (Prasanna et al., 2010). Table 4 lists some examples of begomoviruses re-emerged in Asia in new hosts. Figure 5 shows the geographical distribution of some important begomoviruses in Asia.

**Table 4:** Examples of some important begomoviruses that emerged in new hosts in Asia.

Country	Begomovirus	New host plants	References
China	*Cotton leaf curl Multan virus*	*Gossypium*	Islam et al., 2018
	*Ageratum yellow vein virus*	*Nicotiana tabacum*	Islam et al., 2018
	*Tobacco curly shoot virus*	*Piper nigrum*	Islam et al., 2018
India	*Pepper leaf curl Bangladesh virus*	*Momordica charantia L*	Salati et al., 2010
	*Ageratum enation virus*	*Crassocephalum crepidioides and Ageratum conyzoides*	Yogesh et al., 2011
	*Radish leaf curl virus*	*Abelmoschus esculentus*	Kumar et al., 2012
	*Chili leaf curl virus*	*Datura inoxia*	Marwal et al., 2012
	*Sonchus yellow mosaic virus*	*Jasminum sambac and Millingtonia hortensis*	Marwal et al., 2013
	*Chili leaf curl India virus*	*Mentha spicata*	Saeed et al., 2014
	*Tomato leaf curl New Delhi virus*	*Papaver somniferum*	Srivastava et al., 2016
Indonesia	*Tomato leaf curl New Delhi virus*	*Holothuroidea*	Mizutani et al., 2011
Iran	*Cucurbit chlorotic yellows virus*	*Holothuroidea, Cucumis melo, and Cucurbita*	Bananej et al., 2013
Nepal	*Mungbean yellow mosaic India virus*	*Phaseolus lunatus*	Shahid et al., 2012
Oman	*Chili leaf curl virus*	*Citrullus lanatus*	Shahid et al., 2017
Pakistan	*Tomato leaf curl Palampur virus*	*Momordica charantia*	Ali et al., 2010
	*Squash leaf curl China virus*	*Cucurbita pepo*	Tahir et al., 2010
	*Cotton leaf curl Burewala virus*	*Hibiscus rosa-sinensis*	Akhtar et al., 2014
	*Tomato leaf curl Gujarat virus*	*Gossypium*	Zaidi et al., 2015
	*Tomato leaf curl New Delhi virus*	*Glycine max*	Jamil et al., 2017
	*Alternanthera yellow vein virus*	*Eclipta prostrata*	Zaidi et al., 2017
	*Chickpea chlorotic dwarf virus*	*Abelmoschus esculentus*	Zia-Ur-Rehman et al., 2017
Saudi Arabia	*Tomato chlorosis virus*	*Solanum lycopersicum*	Al-Saleh et al., 2014
	*Watermelon chlorotic stunt virus*	*Citrullus lanatus*	Al-Saleh et al., 2014
Sri Lanka	*Okra yellow vein mosaic virus*	*Abelmoschus esculentus*	Tharmila et al., 2017
South Korea	*Euphorbia leaf curl virus*	*Carica papaya*	Kil et al., 2016

**Figure 5:** Geographical location: The map shows the distribution of some important begomoviruses in Asia.

### Asia: a geographically diverse region for emerging begomoviruses

Several begomoviruses have emerged in Asian countries, including TYLCKaV in Thailand, Tomato yellow leaf curl Indonesia virus, Pepper yellow leaf curl Indonesia virus (PepYLCIV), and Papaya leaf curl virus (PaLCuV). These begomoviruses cause substantial economic losses in Asian countries and increase their host range through mutation and recombination. Brief descriptions of some emerging begomoviruses that are not widely known but very destructive are given below. Figures 6, 7 show the symptoms and phylogenetic analysis, respectively, of these emerging viruses.

**Figure 6:** Symptoms of begomoviruses: **(A)** Tomato plant depicts the symptoms of *Tomato yellow leaf curl Kanchanaburi virus*; **(B)** symptoms of *Pepper yellow leaf curl Indonesia virus*; **(C)** papaya plants exhibit symptoms like yellowing, downward or upward curling, and vein thickening caused by *Papaya leaf curl virus*; **(D)** symptomatic eggplant showing leaf curling caused by *Tomato leaf curl Joydebpur virus*; **(E)** plant showing symptoms of *Tomato yellow leaf curl Thailand virus*; and **(F)** *Tomato yellow leaf curl virus* causes symptoms like leaf yellowing, upward and downward leaf curling, and reduction in leaf size.

**Figure 7:** Phylogeny of DNA-A: The DNA-A sequences of different endemic begomoviruses were downloaded and assembled by Muscle Alignment module in MEGA-11. The phylogeny was constructed by maximum likelihood method with 500 bootstrap replications. The resulting tree was exported and visualized in iTOL (Letunic and Bork, 2021).

### Tomato yellow leaf curl Kanchanaburi virus

TYLCKaV is a bipartite begomovirus with a large host range identified in Thailand’s pepper plants. Resistance and pathogenic determinants in host plants of TYLCKaV have been studied less extensively than those of TYLCV (An et al., 2021). TYLCKaV predominantly infects *Capsicum* species*, Solanum melongena,* and *Solanum lycopersicum.* The spread of TYLCKaV can be reduced using simple procedures, such as isolating greenhouses for transplant production from outdoor sources of begomoviruses. The destruction of whitefly populations is another key management method that might be beneficial for controlling the spread of TYLCKaV (Díaz-Pendón et al., 2010). Figure 6A depicts the symptoms exhibited by TYLCKaV infection.

### Pepper yellow leaf curl Indonesia virus

PepYLCIV is a bipartite begomovirus in which DNA-A and DNA-B play significant roles in infected plants (Fondong, 2013). PepYLCIV was first detected in Central Java in 2003 and was found to infect *Capsicum annuum* (chili peppers) on Sumatra Island in 2005 (De Barro et al., 2008). Chili peppers are largely grown in Indonesia to meet the strong market demand. This crop has recently been decimated in Indonesia due to PepYLCIV infection (Fondong, 2013). This pathogen can infect hot peppers, sweet peppers, tomatoes, and weeds, causing symptoms such as leaf curling, yellowing in young leaves, and stunting (Fadhila et al., 2020). Figure 6B depicts the symptoms of PepYLCIV in chili fields and plants.

### Papaya leaf curl virus

PaLCuV is a monopartite begomovirus and is transmissible through *B. tabaci* on a wide range of hosts. It can infect *Carica papaya L* (papaya), *Cestrum nocturnum, Capsicum* species, *Cyamopsis tetragonoloba*, *Nicotiana tabacum*, and *S. lycopersicum* (Lal et al., 2020). It causes one of the most severe viral diseases affecting papaya crops in tropical areas. Infected papaya plants exhibit symptoms, such as yellowing, downward, or upward curling, and vein thickening, whereas severely infected plants have curled petioles and wilting (Varun et al., 2017). Symptoms can be seen in Figure 6C. Currently, the most common treatments used to control the spread of PaLCuV include an extensive range of insecticides and crop rotation. Removing the infected plants and destroying infected fields are also performed to avoid the disease spread.

### Tomato leaf curl Joydebpur virus

ToLCJoV is a monopartite virus that poses a significant threat to tomato production in eastern India. ToLCJoV was first identified in Bangladesh by Maruthi et al. (2005). It infects chili and *Hibiscus cannabinus* (kenaf) worldwide (Paul et al., 2009). The virus is transmitted only by whiteflies (Paul et al., 2009). ToLCJoV can infect *S. lycopersicum*, *Capsicum frutescens*, *Phaseolus vulgaris, Solanum nigrum, Amaranthus viridis, Hibiscus cannabinus,* and *S. melongena* globally, causing symptoms such as vein clearing, leaf curling, decrease in leaf lamina, vein enation, and stunting Figure 6D (Hamim et al., 2020).

### Tomato yellow leaf curl Thailand virus

TYLCTHV (Genus: *Begomovirus*, Family: *Geminiviridae*) has a monopartite genome that contains a single molecule of circular ssDNA (DNA-A). *Bemisia tabaci* is responsible for its transmission. The major symptoms of TYLCTHV infection are leaf curling and yellowing (Khan et al., 2012). The virus was first reported in Thailand in 1994 (Blawid et al., 2008) and has now dispersed to Myanmar (Green et al., 2001), South China (Guo et al., 2009), and was recently identified in Taiwan in 2005 (Jan et al., 2007). As a prominent tomato-infecting begomovirus, TYLCTHV alters the dynamics of pre-tomato begomoviruses and adversely affects Taiwan’s tomato production. TYLCTHV is probably more pathogenic and invasive, with a broad host range, and it outlasts and substitutes *Tomato yellow leaf curl Taiwan virus*, possibly due to more efficient transmission by indigenous or introduced whitefly biotypes (Tsai et al., 2011). Figure 6E shows symptoms produced by TYLCTHV in tomato.

## Discussion

Begomovirus disease complexes are rapidly growing in terms of geographical distribution and host range. For example, TYLCV is spreading to new areas in the Indian and Pacific regions, including New Caledonia, Australia, and Mauritius (Mabvakure et al., 2016). Before 2010, ToLCNDV was only limited to Asia but now it has been spread throughout Europe and has increased its host plant range, including *Euphorbiaceae*, *Cucurbitaceae*, *Fabaceae*, and *Malvaceae* (Moriones et al., 2017). Similarly, CMD has been widespread in Africa until 2015, when SLCMV was spread in Southeast Asia (Wang et al., 2016).

The presence of multiple hosts and expansion in the whitefly population around the globe has contributed to the spread of the begomoviruses. With the existence of such a wide population of begomoviruses along with their ability to exchange genetic material through recombination, new begomoviruses have also been emerging has the potential to spread as a pandemic. In addition to the evolution, human beings also played a significant role in the spread of begomovirus diseases in different ways, such as moving crops from their original location to another environment or through germplasm transfer to a different environment (Seal et al., 2006).

This review highlighted the introduction of emerging begomoviruses in Asia that have potential to spread as pandemic. We also highlighted currently less important endemic viruses: TYLCKaV, PepYLCIV, PaLCuV, ToLCJoV, and TYLCTHV. The factors driving the emergence of plant viruses include global movement of plant materials and increase in the population of insect vectors. Another aspect involved in begomovirus outbreaks is the connection of complex viruses with betasatellites. Given the alarming rate at which novel begomoviruses are appearing in tomato, peppers, papaya, eggplant, chili and other crops, there is always an urgent need to create economic and ecologically appropriate strategies for successful virus control.

### Future perspectives

Recent developments highlight the diversity in host ranges of begomoviruses with strong evidence indicating that an increasing number of host species reported with time in different regions in the world. It is envisioned to properly investigate the Intra- and inter-regional diversification of begomoviruses with applying preventive measures to control their transmission. Moreover, certain aspects i.e., associated satellite molecules with unique properties particularly those related to the specific morphological changes caused by infection, begomovirus interaction with insect vectors and transmission methodology adopted by begomoviruses would give an additional approach to investigating begomoviruses. It is the collective responsibility of the scientific community to develop a thorough plan and policy to counteract this before a devastating effect on food security and the global economy is realized.

## Author contributions

MQ, AL, E-JK, and SL outlined and conceptualized the review theme. MQ wrote the first draft of the manuscript. BN, TV, GS, PH, E-JK, SJ, K-YL, C-WT, HD, TH, T-TA, NW, JL, S-MK, MN-u-R, and SL contributed to the manuscript preparation and revision, and also read and approved the submitted version. All authors contributed to the article and approved the submitted version.

## Funding

This work was supported by the Research Program (Grant #Z-1543086-2017-21-01 and Grant # B-1543086-2021-23) for the Exportation Support of Agricultural Products at the Animal and Plant Quarantine Agency of the Republic of Korea.

## Conflict of interest

JL was employed by company NongWoo Bio.

The remaining authors declare that the research was conducted in the absence of any commercial or financial relationships that could be construed as a potential conflict of interest.

## Publisher’s note

All claims expressed in this article are solely those of the authors and do not necessarily represent those of their affiliated organizations, or those of the publisher, the editors and the reviewers. Any product that may be evaluated in this article, or claim that may be made by its manufacturer, is not guaranteed or endorsed by the publisher.
